RETRACTED

# A kinase‐interacting protein 1 may serve as a potential biomarker for deteriorative tumor features and poor prognosis in gastric cancer patients

**DOI:** 10.1002/jcla.23350

**Published:** 2020-07-16

**Authors:** Rongbo Lin, Shen Zhao, Liyu Su, Xiaohui Chen, Chunwei Xu, Qinliang He, Changhua Zhuo, Yunbin Ye

**Affiliations:** ^1^ Department of Gastrointestinal Medical Oncology Fujian Cancer Hospital & Fujian Medical University Cancer Hospital Fuzhou China; ^2^ Fujian Key Laboratory of Translational Cancer Medicine Fuzhou China; ^3^ Department of Thoracic Surgery Fujian Cancer Hospital & Fujian Medical University Cancer Hospital Fuzhou China; ^4^ Department of Pathology Fujian Cancer Hospital & Fujian Medical University Cancer Hospital Fuzhou China; ^5^ Department of Gastrointestinal Surgical Oncology Fujian Cancer Hospital & Fujian Medical University Cancer Hospital Fuzhou China; ^6^ Laboratory of Immuno‐Oncology Fujian Cancer Hospital & Fujian Medical University Cancer Hospital Fuzhou China

**Keywords:** A kinase‐interacting protein 1, clinicopathological characteristics, disease‐free survival, gastric cancer, overall survival

## Abstract

**Objective:**

This study aimed to explore the association of A kinase‐interacting protein 1 (AKIP1) expression with clinicopathological characteristics and prognosis in gastric cancer patients.

**Methods:**

Data of 260 gastric cancer patients were retrospectively reviewed. AKIP1 expression in tumor tissue and non‐cancerous tissue specimens was detected by immunohistochemistry and semi‐quantitatively scored according to the staining intensity and density. Moreover, the clinicopathological features were retrieved, and disease‐free survival (DFS) and overall survival (OS) were calculated.

**Results:**

A kinase‐interacting protein 1 expression was increased in tumor tissues compared with non‐cancerous tissues (*P* < .001). In terms of tumor features, tumor AKIP1 high expression correlated with elevated T stage (*P* < .001) and raised TNM stage (*P* = .042), while did not correlate with pathological grade (*P* > .999), tumor size (*P* = .060), N stage (*P* = .180), or tumor location (*P* > .999). Meanwhile, tumor AKIP1 was not associated with the non‐tumor features either. Kaplan‐Meier curves disclosed that AKIP1 high expression patients had shorter DFS (*P* = .004) and OS (*P* = .043) compared with AKIP1 low expression patients. Univariate Cox's regression showed that AKIP1 high expression correlated with shorter DFS (*P* = .005, hazard ratio [HR] = 1.635) and OS (*P* = .046, HR = 1.519), whereas multivariate Cox's regression displayed that AKIP1 did not independently predict worse DFS (*P* = .172, HR = 1.276) or shorter OS (*P* = .433, HR = 1.183).

RETRACTED

**Conclusion:**

A kinase‐interacting protein 1 may serve as a potential biomarker for deteriorative tumor features and poor prognosis in gastric cancer patients.

## 1 INTRODUCTION

Gastric cancer remains the fifth most common cancer globally and is the third most common cause of cancer death worldwide.^1^, ^2^, ^3^ Despite the progresses in detection methods, surgical technology, and medicine therapies in these years and the 5‐year survival rate of early gastric cancer can reach >90%, most patients present with advanced‐stage gastric cancer, which limited treatment options, and the global 5‐year survival rate is 5%‐10% in advanced stages.^3^, ^4^, ^5^, ^6^, ^7^ Thus, the management of gastric cancer is challenging. Identifying convincing biomarkers for prognosis may offer insights into prognostication and contribute to development of individualized treatment strategies in gastric cancer patients.

A kinase‐interacting protein 1 (AKIP1), a small 23‐kDa protein, is initially discovered in breast cancer cells and reported to facilitate the nuclear translocation of catalytic subunit of protein kinase A.^8^ Recent studies have indicated that AKIP1 is dysregulated in various human malignancies and may represent the physiological or pathological abnormities.^9^, ^10^, ^11^, ^12^ For instance, AKIP1 has been found overexpressed in tumor tissues of breast cancer, non‐small‐cell lung cancer, and colorectal mucosa, and its upregulated expression correlates with advanced disease progression and worse overall survival (OS) in these cancers.^9^, ^10^, ^11^, ^12^ For the role of AKIP1 in gastric cancer, just one literature shows that AKIP1 promotes cell proliferation, migration, invasion via inducing Slug‐mediated epithelial‐mesenchymal transition (EMT) and correlates with poor prognosis in gastric cancer, whereas the small sample size of 96 patients limits its value in clinical settings.^11^ Hence, in this present study, we detected AKIP1 expression in 260 surgical gastric cancer patients and aimed to explore the association of AKIP1 expression with clinicopathological characteristics and prognosis in gastric cancer patients.

## 2 MATERIALS AND METHODS

### 2.1 Patients

This retrospective study reviewed 260 gastric cancer patients who were screened from our hospital database. All patients received resection in our hospital between July 2014 and June 2017. Patients were eligible for analysis in the current study if they initially diagnosed as primary gastric cancer, with age between 18 and 80 years, had well preserved tumor tissue and non‐cancerous tissue as well as complete preoperative tumor features and follow‐up data, without neoadjuvant therapy. Notably, the definitions of some clinical characteristics were as follows: hypertension was defined as a history of high blood pressure (≥140/90 mm Hg) reported by the respondent or current use of antihypertensive medication; hyperlipidemia was defined as current use of antilipidemic medication, TC ≥ 5.70 mmol/L, serum TGs ≥ 1.70 mmol/L, or LDL‐C ≥ 3.10 mmol/L; diabetes mellitus was defined as a previous diagnosis, treatment with insulin or oral hypoglycemic medications, fasting plasma glucose ≥126 mg/dL, or glycosylated hemoglobin ≥6.5%.^13^, ^14^ This study was approved by the Institutional Review Board of our hospital. All patients or their family members provided written informed consents before enrollment.

RETRACTED

### 2.2 Immunohistochemistry (IHC) staining

Tumor tissue and non‐cancerous tissue specimens were obtained from Pathology department of our hospital, and all tissue specimens were formalin‐fixed and paraffin‐embedded. The non‐cancerous tissues of gastric cancer patients were the cancer‐adjacent normal tissues >5 cm away from the tumor. The expression of AKIP1 in tissue specimen was detected by IHC. The procedures were carried out as follows: firstly, the tissue specimens were cut into 4 μm sections; then, all sections were deparaffinized, rehydrated, and antigen retrieval; subsequently, 10% normal goat serum (Sigma‐Aldrich) was added following peroxidase activity was blocked; after that, Rabbit polyclonal to C11orf17 (1:100, Abcam) was added and incubated at 4°C overnight; the next day, horseradish peroxidase‐conjugated Goat anti‐Rabbit IgG (H + L) Secondary Antibody (1:10 000, Thermo Fisher) was added and incubated at 37°C for 60 minutes; finally, the sections were stained, counterstained, and sealed.

### 2.3 IHC assessment

The result of IHC staining was observed using Nikon ECLIPSE E200 microscope (Nikon Instruments) and assessed based on staining intensity and proportion of positively stained cells.^15^ Briefly, 5 high‐power fields were selected for evaluating the score of staining intensity and density. The staining intensity was scored as follows: 0, no staining; 1, weak staining; 2, moderate staining; and 3, strong staining. A hundred cells in the 5 high‐power fields were counted for assessing staining density, which was calculated by the positively stained cells proportion. The staining density was scored as follows: 0, no positively stained cells; 1, 1%‐25% of positively stained cells; 2, 26%‐50% of positively stained cells; 3, 51%‐75% of positively stained cells; and 4, 76%‐100% of positively stained cells. The total IHC score was calculated through the staining intensity score multiplied by the staining density score. AKIP1 high expression was defined as total IHC score ≥3, and AKIP1 low expression was defined as the total IHC score <3.

RETRACTED

### 2.4 Follow‐up

According to the document of follow‐up data, the median follow‐up duration was 34.0 months with the last follow‐up date of 2019/06/30. And the minimum and maximum of follow‐up duration was 4.0 months and 60.0 months, respectively. Disease‐free survival (DFS) was defined as the duration from resection to disease relapse, disease progression, or death, and overall survival (OS) was defined as the duration from resection to death.

### 2.5 Statistical analysis

Statistical analyses were performed using SPSS version 22.0 (IBM), and figures were plotted using GraphPad Prism version 7.00 (GraphPad Software). Descriptive statistics were displayed as mean ± standard deviation (SD) for continuous variables and count (percentage) for categorical variables. Comparison of AKIP1 expression between tumor tissue and non‐cancerous tissue was determined by McNemar's test. Correlation of AKIP1 expression with pathological grade, tumor size, T stage, N stage, TNM stage, or tumor location was determined by Wilcoxon's rank sum test or chi‐square test and corrected by Bonferroni test. Correlation of AKIP1 expression with demographics, complications, *Helicobacter pylori* infection, or tumor location was analyzed by chi‐square test. DFS and OS were displayed using Kaplan‐Meier curve, and comparison of DFS or OS between AKIP1 high expression and AKIP1 low expression patients was determined by log‐rank test. Factors predicting DFS and OS were analyzed by univariate Cox's regression, and variables that achieved statistical significance at *P* < .05 in univariate Cox's regression were further included in the multivariate Cox's proportional hazard regression model. *P* value <.05 was considered as significant.

## 3 RESULTS

### 3.1 Study flow

Four hundred and fifty‐one gastric cancer patients who underwent resection were screened in our study, while 191 patients were excluded, including 83 patients who received neoadjuvant therapy, 69 patients who were unable to obtain informed consents, 25 patients who were with unavailable tumor tissues or non‐cancerous tissues, 10 patients who had incomplete clinicopathological tumor features or incomplete relapse, relapse, progression, and survival data, and 4 patients who were with secondary or relapsed gastric cancer (Figure 1). Then, the remaining 260 gastric cancer patients were reviewed in this study, and their clinicopathological and follow‐up data were collected. Additionally, their tumor and non‐cancerous tissue specimens were obtained, and AKIP1 expression was detected by IHC. All 260 patients were included in final analysis.

RETRACTED

**Figure 1:** Study flow

### 3.2 Clinicopathological characteristics of gastric cancer patients

The mean age (including 112 [43.1%] females and 148 [56.9%] males) was 59.2 ± 11.2 years (Table 1). Besides, there were 81 (31.2%), 88 (33.8%), 83 (31.9%), 73 (28.1%), 40 (15.4%), and 93 (35.8%) patients had current smoke, current drink, hypertension, hyperlipidemia, diabetes, and *H pylori* infection, respectively. For tumor features, 67 (25.8%), 28 (10.8%), and 165 (63.4%) patients presented with tumor in cardia, tumor in gastric body, and tumor in gastric antrum, respectively; 34 (13.1%), 187 (71.9%), and 39 (15.0%) patients presented with pathological grade G1, G2, and G3, respectively; mean tumor size was 3.2 ± 1.2 cm; 7 (2.7%), 18 (6.9%), 233 (89.6%), and 2 (0.8%) patients were with T1 stage, T2 stage, T3 stage, and T4 stage, respectively; 73 (28.1%), 62 (23.8%), 107 (41.2%), and 18 (6.9%) patients showed N0 stage, N1 stage, N2 stage, and N3 stage, respectively; 25 (9.6%), 107 (41.2%), and 128 (49.2%) patients presented with TNM stage Ⅰ, TNM stage Ⅱ, and TNM stage III, respectively. As for the post‐surgery treatments, 172 (66.2%) patients received adjuvant chemotherapy and 35 (13.5%) patients received adjuvant radiotherapy, respectively.

**Table 1:** Clinicopathological characteristics

Items	Gastric cancer patients (N = 260)
Age (y), mean ± SD	59.2 ± 11.2
Gender, No. (%)	
Female	112 (43.1)
Male	148 (56.9)
Current smoke, No. (%)	
No	179 (68.8)
Yes	81 (31.2)
Current drink, No. (%)	
No	172 (66.2)
Yes	88 (33.8)
Hypertension, No. (%)	
No	177 (68.1)
Yes	83 (31.9)
Hyperlipidemia, No. (%)	
No	187 (71.9)
Yes	73 (28.1)
Diabetes, No. (%)	
No	220 (84.6)
Yes	40 (15.4)
*Helicobacter pylori* infection, No. (%)	
Negative	167 (64.2)
Positive	93 (35.8)
Tumor location, No. (%)	
Cardia	67 (25.8)
Gastric body	28 (10.8)
Gastric antrum	165 (63.4)
Pathological grade, No. (%)	
G1	34 (13.1)
G2	187 (71.9)
G3	39 (15.0)
Tumor size (cm), mean ± SD	3.2 ± 1.2
T stage, No. (%)	
T1	7 (2.7)
T2	18 (6.9)
T3	233 (89.6)
T4	2 (0.8)
N stage, No. (%)	
N0	73 (28.1)
N1	62 (23.8)
N2	107 (41.2)
N3	18 (6.9)
TNM stage, No. (%)	
I	25 (9.6)
II	107 (41.2)
III	128 (49.2)
Adjuvant chemotherapy, No. (%)	
No	88 (33.8)
Yes	172 (66.2)
Adjuvant radiotherapy, No. (%)	
No	225 (86.5)
Yes	35 (13.5)

Abbreviation: SD, standard deviation.

### 3.3 Comparison of AKIP1 expression between tumor tissue and non‐cancerous tissue in gastric cancer patients

Immunohistochemistry was applied to detect AKIP1 expression in tumor tissue and non‐cancerous tissue, and the examples of AKIP1 expression were displayed in Figure 2A. We found that AKIP1 expression was increased in tumor tissues compared with non‐cancerous tissues (*P* < .001) (Figure 2B).

RETRACTED

**Figure 2:** AKIP1 expressions in tumor tissue and non‐cancerous tissue. Examples of AKIP1 expression by IHC detection (A). Comparison of AKIP1 expression between tumor tissue and non‐cancerous tissue (B). AKIP1, A kinase‐interacting protein 1; IHC, immunohistochemistry

### 3.4 Correlation of tumor AKIP1 expression with clinicopathological features in gastric cancer patients

In terms of tumor features, no correlation of tumor AKIP1 expression with pathological grade (*P* > .999) (Figure 3A), tumor size (*P = *.060) (Figure 3B), N stage (*P* = .180) (Figure 3D), or tumor location (*P* > .999) (Figure 3F) was observed, whereas tumor AKIP1 high expression was associated with elevated T stage (*P* < .001) (Figure 3C) and raised TNM stage (*P* = .042) (Figure 3E). As to clinical characteristics apart from tumor features, no correlation of AKIP1 expression with age (*P* = .323), gender (*P* = .646), current smoke (*P* = .332), current drink (*P* = .880), hypertension (*P* = .144), hyperlipidemia (*P* = .609), diabetes (*P* = .285), or H. pylori infection (*P* = .389) was observed in gastric cancer patients (Table S1).

**Figure 3:** Association of tumor AKIP1 expression with tumor features. Association of tumor AKIP1 expression with pathological grade (A). Association of tumor AKIP1 expression with tumor size (B). Association of tumor AKIP1 expression with T stage (C). Association of tumor AKIP1 expression with N stage (D). Association of tumor AKIP1 expression with TNM stage (E). Association of tumor AKIP1 expression with tumor location (F). AKIP1, A kinase‐interacting protein 1

### 3.5 Correlation of tumor AKIP1 expression with DFS and OS in gastric cancer patients

A total of 143 patients relapsed, and 98 patients died in this study. DFS in patients with AKIP1 high expression was shorter than that in patients with AKIP1 low expression (*P* = .004) (Figure 4A); meanwhile, OS in patients with AKIP1 high expression was also decreased than that in patients with AKIP1 low expression (*P* = .043) (Figure 4B).

**Figure 4:** Survival profiles. DFS in AKIP1 high expression patients and AKIP1 low expression patients (A). OS in AKIP1 high expression patients and AKIP1 low expression patients (B). DFS, disease‐free survival; AKIP1, A kinase‐interacting protein 1; OS, overall survival

### 3.6 Analysis of factors affecting DFS in gastric cancer patients

Univariate Cox's regression showed that tumor AKIP1 high expression was associated with reduced DFS (*P* = .005, hazard ratio [HR]: 1.635 [95% confidence interval [CI]: 1.163‐2.299]); meanwhile, higher pathological grade (*P* < .001, HR: 2.502 [95%CI: 1.836‐3.408]) and higher TNM stage (*P* < .001, HR: 1.931 [95%CI: 1.462‐2.550]) were associated with poorer DFS in gastric cancer patients, as well (Table 2). Furthermore, multivariate analysis displayed that tumor AKIP1 high expression (*P* = .172, HR: 1.276 [95%CI: 0.899‐1.812]) did not independently predict worse DFS, while higher pathological grade (*P* < .001, HR: 2.197 [95%CI: 1.603‐3.011]) and higher TNM stage (*P* < .001, HR: 1.655 [95%CI: 1.248‐2.193]) were independent predictive factors for worse DFS.

RETRACTED

**Table 2:** Analysis of factors affecting DFS

Items	Cox's proportional hazard regression model	
	*P* value	HR (95%CI)
Univariate Cox's regression		
AKIP1 high expression	.005	1.635 (1.163‐2.299)
Age (>60 y)	.490	0.891 (0.642‐1.237)
Gender (male)	.455	1.136 (0.813‐1.586)
Current smoke	.336	0.837 (0.584‐1.202)
Current drink	.877	0.973 (0.688‐1.377)
Hypertension	.343	0.841 (0.588‐1.203)
Hyperlipidemia	.243	1.236 (0.866‐1.763)
Diabetes	.921	0.977 (0.620‐1.540)
*Helicobacter pylori* positive	.579	1.101 (0.784‐1.547)
Tumor location		
Gastric antrum	Reference	—
Cardia	.449	1.159 (0.791‐1.697)
Gastric body	0.168	1.431 (0.860‐2.379)
Higher pathological grade	<.001	2.502 (1.836‐3.408)
Higher TNM stage	<.001	1.931 (1.462‐2.550)
Adjuvant chemotherapy	.996	1.001 (0.704‐1.422)
Adjuvant radiotherapy	.576	1.145 (0.713‐1.837)
Multivariate Cox's regression		
AKIP1 high expression	.172	1.276 (0.899‐1.812)
Higher pathological grade	<.001	2.197 (1.603‐3.011)
Higher TNM stage	<.001	1.655 (1.248‐2.193)

Note

The factors with *P* < .05 in the univariate Cox's regression were included in the multivariate Cox's regression.

Abbreviations: AKIP1, A kinase‐interacting protein 1; CI, confidence interval; DFS, disease‐free survival; HR, hazard ratio.

### 3.7 Analysis of factors affecting OS in gastric cancer patients

In regard to factors affecting OS in gastric cancer patients, the univariate analysis disclosed that tumor AKIP1 high expression (*P* = .046, HR: 1.519 [95%CI: 1.008‐2.289]) was correlated with worse OS, and higher pathological grade (*P* < .001, HR: 2.440 [95%CI: 1.674‐3.558]) and higher TNM stage (*P* < .001, HR: 2.077 [95%CI: 1.459‐2.958]) also correlated with decreased OS in gastric cancer patients (Table 3). The multivariate analysis showed that AKIP1 high expression (*P* = .433, HR: 1.183 [95%CI: 0.777‐1.801]) was not an independent predictive factor, but higher pathological grade (*P* < .001, HR: 2.088 [95%CI: 1.418‐3.073]) and higher TNM stage (*P* = .002, HR: 1.766 [95%CI: 1.233‐2.528]) independently predicted shorter OS (Table 3). These data implied that tumor AKIP1 might predict OS through affecting TNM stage in gastric cancer patients.

RETRACTED

**Table 3:** Analysis of factors affecting OS

Items	Univariate Cox's regression	
	*P* value	HR (95%CI)
Univariate Cox's regression		
AKIP1 high expression	.046	1.519 (1.008‐2.289)
Age (>60 y)	.927	0.982 (0.660‐1.459)
Gender (male)	.391	1.195 (0.796‐1.794)
Current smoke	.364	0.816 (0.526‐1.266)
Current drink	.490	0.861 (0.562‐1.318)
Hypertension	.059	0.641 (0.404‐1.016)
Hyperlipidemia	.550	1.141 (0.739‐1.762)
Diabetes	.806	0.932 (0.529‐1.641)
*Helicobacter pylori* positive	.749	1.069 (0.709‐1.613)
Tumor location		
Gastric antrum	Reference	—
Cardia	.125	1.422 (0.907‐2.230)
Gastric body	.076	1.702 (0.946‐3.064)
Higher pathological grade	<.001	2.440 (1.674‐3.558)
Higher TNM stage	<.001	2.077 (1.459‐2.958)
Adjuvant chemotherapy	.884	0.969 (0.635‐1.479)
Adjuvant radiotherapy	.388	1.275 (0.735‐2.212)
Multivariate Cox's regression		
AKIP1 high expression	.433	1.183 (0.777‐1.801)
Higher pathological grade	<.001	2.088 (1.418‐3.073)
Higher TNM stage	.002	1.766 (1.233‐2.528)

Note

The factors with *P* < .05 in the univariate Cox's regression were included in the multivariate Cox's regression.

Abbreviations: AKIP1, A kinase‐interacting protein 1; CI, confidence interval; HR, hazard ratio; OS, overall survival.

## 4 DISCUSSION

A kinase‐interacting protein 1, localizing in cytoplasm, nucleus, and mitochondria, functions as an adaptor of structural intracellular protein.^16^ Recently, AKIP1 has been shown to facilitate tumorigenesis and invasiveness.^9^, ^10^, ^11^, ^12^ For example, one study displays that AKIP1 promotes cell migration, invasion, and EMT through mediating transactivating Zinc Finger E‐Box Binding Homeobox 1 (ZEB1) in non‐small‐cell lung cancer cells.^9^ Besides, an experiment shows that AKIP1 downregulation represses cell motility and invasion via suppressing the Akt/glycogen synthase kinase (GSK)‐3β/Snail pathway in breast cancer cells.^10^ Additionally, a study discloses that AKIP1 promotes angiogenesis via upregulating the nuclear factor kappa‐B (NF‐κB) dependent chemokine C‐X‐C motif ligand (CXCL) 1, CXCL2, and CXCL8 in cervical cancer cells.^17^ For gastric cancer, a previous study displays that AKIP1 enhances gastric cancer cell proliferation, migration and invasion via activating Slug‐induced EMT.^11^ These data reveal that AKIP1 may promote cell proliferation, migration, and invasion, which contributes to its function as an oncogenic factor in the pathology of specific cancers, including gastric cancer.

Apart from these experiments, some studies have uncovered the role of AKIP1 in clinical practices of cancers.^9^, ^10^, ^11^, ^12^ For instance, AKIP1 is overexpressed in breast cancer tissues and colorectal mucosa tissues.^10^, ^12^ Moreover, AKIP1 is found to be upregulated in non‐small‐cell lung cancer patients, and its expression is positively associated with TNM stage and lymph node metastasis in these patients.^9^ Also, AKIP1 high expression is associated with advanced tumor stage, larger tumor size, and presence of lymph node metastasis in breast cancer patients.^10^ Additionally, AKIP1 expression positively associates with TNM stage, tumor diameter, and lymph node metastasis in colorectal cancer patients.^12^ These data imply that AKIP1 may be overexpressed and positively associated with disease progression in specific cancers. As to gastric cancer, there is only one study that displays the correlation of AKIP1 overexpression with poor prognosis in gastric cancer patients, while sample size in that previous study (N = 96) is small, resulting in insufficient statistical power and limited clinical significance, and the correlation of AKIP1 with clinicopathological characteristics as well as prognosis of gastric cancer need further investigation. To solve this problem, we retrospectively assessed the data of 260 surgical gastric cancer patients and detected their AKIP1 expressions. Subsequently, we found that AKIP1 expression was dramatically increased in tumor tissues than that in non‐cancerous tissues, which might be due to the following fact: AKIP1 interacted with Slug to facilitate the malignant proliferation of gastric cancer cells, and thereby promoting the tumor occurrence, thus, AKIP1 expression was overexpressed in tumor tissues compared with non‐cancerous tissues in gastric cancer patients.^11^ Furthermore, we explored the association of AKIP1 expression with clinicopathological characteristics in gastric cancer patients and observed that AKIP1 high expression was correlated with increased T stage and higher TNM stage in gastric cancer patients. The possible reasons were as follows: (a) AKIP1 probably not only promoted cell proliferation via activating Slug‐induced EMT, but also promoted angiogenesis via increasing NF‐κB dependent CXCL1, CXCL2, and CXCL8 levels, which facilitated the tumor growth of gastric cancer, resulting in the positive correlation of AKIP1 expression with T stage and TNM stage in gastric cancer patients ^11^, ^17^; (b) similar to its influence in other cancer cells, AKIP1 might activate ZEB1 or regulate Akt/GSK‐3β/Snail pathway to promote cell migration and invasion of gastric cancer cells, leading to the lymphatic metastasis; therefore, AKIP1 high expression was associated with elevated TNM stage in gastric cancer patients.^9^, ^10^

As to the prognostic value of AKIP1 in gastric cancer, previous studies have shown that AKIP1 high expression is associated with poor DFS in non‐small‐cell lung cancer patients and also correlates with worse OS in breast cancer patients and colorectal cancer patients.^9^, ^10^, ^12^ In the present study, we found that AKIP1 expression was negatively associated with DFS and OS in gastric cancer patients. These results might be account of that (a) AKIP1 might promote cell proliferation, repress apoptosis, and enhance angiogenesis via activating some related proteins (ZEB1 or Slug) to aggravate disease progression, thereby leading to poor DFS and OS in gastric cancer patients ^9^, ^10^, ^11^; (b) AKIP1 might reduce the chemotherapy sensitivity of gastric cancer cells; for instance, one previous study reveals that AKIP1 correlates with increased chemotherapy resistance in serous ovarian cancer, and thus, it decreased treatment efficacy and eventually resulted in worse DFS and OS in gastric cancer patients, while detailed mechanism in gastric cancer was elusive.^18^ Moreover, we observed that was not an independent predictive factor for worse DFS or OS, implying that AKIP1 might predict DFS or OS via affecting other independent predictive factors (such as TNM stage) in gastric cancer patients.

RETRACTED

There were still some limitations in our study. Firstly, the median follow‐up duration (34.0 months) was relatively short, and association of AKIP1 expression with prognosis of gastric cancer patients in long term needs further exploration; Secondly, the underlying mechanism of AKIP1 in gastric cancer remained unclear, which was necessary to be investigated in further studies; Thirdly, this was a retrospective study and the AKIP1 expression was restricted to IHC, and thus, further prospective study with other tools (such as qPCR) was needed to validate our results.

To conclude, AKIP1 is overexpressed in tumor tissues compared with non‐cancerous tissues; meanwhile, tumor AKIP1 high expression correlates with deteriorative tumor features and predicts worse survival profiles in gastric cancer patients, which imply that AKIP1 may serve as a potential biomarker for advanced progression and poor prognosis of gastric cancer.

## Supporting information

Table S1
